# HIF-1α and HIF-2α: Siblings in Promoting Angiogenesis of Residual Hepatocellular Carcinoma after High-Intensity Focused Ultrasound Ablation

**DOI:** 10.1371/journal.pone.0088913

**Published:** 2014-02-13

**Authors:** Lun Wu, Zhihao Fu, Shiji Zhou, Jianping Gong, Chang An Liu, Zhengrong Qiao, Shengwei Li

**Affiliations:** 1 The Department of Hepatobiliary Surgery, The Second Affiliated Hospital of Chongqing Medical University, Chongqing Key Laboratory of Hepatobiliary Surgery, Chongqing, China; 2 The Department of Gastrointestinal Surgery, The Second Affiliated Hospital of Chongqing Medical University, Chongqing, China; 3 The Department of General Surgery, The People’s Five Hospital of Chongqing, Chongqing, China; University of Hawaii Cancer Center, United States of America

## Abstract

**Background:**

High-intensity focused ultrasound (HIFU) is a widely applied to treatment for unresectable hepatocellular carcinoma. However, insufficient HIFU can result in rapid progression of the residual tumor. The mechanism of such rapid growth of the residual tumor after HIFU ablation is poorly understood.

**Objective:**

The aim of this study was to investigate the dynamic angiogenesis of residual tumor, and the temporal effect and mechanism of the HIF-1, 2α in the residual tumor angiogenesis.

**Methods:**

Xenograft tumors of HepG2 cells were created by subcutaneously inoculating nude mice (athymic BALB/c nu/nu mice) with hepatoma cells. About thirty days after inoculation, all mice (except control group) were treated by HIFU and assigned randomly to 7 groups according to various time intervals (1st, 3rd, 5th day (d) and 1st, 2nd, 3rd, 4th week (w)). The residual tumor tissues were obtained from the experimental groups at various time points. Protein levels of HIF-1α, HIF-2α, VEGF-A, and EphA2 were quantified by immunohistochemistry analysis and Western Blot assays, and mRNA levels measured by Q-PCR. Microvascular density was calculated with counting of CD31 positive vascular endothelial cells by immunohistochemical staining.

**Results:**

Compared with the control group, protein and mRNA levels of HIF-1α reached their highest levels on the 3rd day (P<0.01), then decreased (P<0.05). HIF-2α expression reached its highest level on the 2nd week compared with control group (P<0.01), then decreased (2w–4w) (P<0.05). The protein and mRNA levels of VEGF-A and EphA2 in the residual tumor tissues group that received HIFU were significantly decreased until 1 week compared with the control group (P<0.01). However, the levels increased compared to controls in 2–4 weeks (P<0.05). Similar results were obtained for MVD expression (P<0.05).

**Conclusion:**

Insufficient HIFU ablation promotes the angiogenesis in residual carcinoma tissue over time. The data indicate that the HIF-1, 2α/VEGFA/EphA2 pathway is involved.

## Introduction

Hepatocellular carcinoma (HCC) is the sixth most common cancer, and the third most common cause of cancer-related death globally. It frequently has features of high malignancy and poor prognosis [1]. However, patients are often diagnosed at an intermediate or advanced stage when few effective therapies are available. With advancement in technologies, local ablation therapies have emerged as effective treatment options. HIFU is considered as a meaningful adjuvant treatment for technically un-resectable HCC, and is an effective, and safe, therapeutic method at present [2]. Unfortunately, even with radical HIFU ablation, residual tumor can appear due to recurrence, and rapid progression of the tumor. This results in clinical deterioration, and poor prognosis. However, the mechanisms by which the rapid growth of residual HCC after HIFU ablation occurs, and the mediators involved are still poorly understood.

Hypoxia inducible factor-1 alpha (HIF-1α), a master regulator of essential adaptive responses to hypoxia, is highly expressed under hypoxic conditions, but maintains a low concentration under normoxic condition [3]. Its levels are generally increased in aggressive tumors [4], and it can be an independent predictor of poor prognosis in HCC [5]. HIF-1α plays a major role in the development of characteristic tumor phenotypes including growth rate, angiogenesis, invasiveness, and metastasis [6]. Angiogenesis plays a particularly important role in tumor formation and maintenance [7]. A great number of angiogenesis-associated genes are directly induced by HIF-1α, such as NOS (nitric oxide synthases), angiogenic and vascular growth factors (VEGF). The vascular endothelial growth factor (VEGF) family of structurally related molecules including VEGFA, VEGFB, VEGFC, VEGFD and placental growth factor (PLGF), is one of the most potent angiogenic factors expressed in various human cancers [8]. Studies have shown that VEGF is frequently expressed in HCC [9]. Hypoxia inducible factor-2 alpha (HIF-2α) is also current focus of research in angiogenesis. The expression of angiogenic genes in hepatocytes is predominantly regulated by HIF-2α, suggesting involvement of HIF-2α in regulating angiogenesis in HCC [10]. Epithelial cell kinase (EphA2) is a member of the Eph family of receptor tyrosine kinases, and highly expressed in many aggressive cancer types, including HCC. It has been found that EphA2 is expressed in tumor cells and endothelial cells in these xenografts, and also in vasculature and tumor cells of surgically removed human cancers [11]. Over-expression of EphA2 is associated with key mediators of angiogenesis and invasion [12].

We hypothesized that insufficient HIFU ablation could result in angiogenesis and proliferation of residual HCC, and play a key role in the rapid growth of residual HCC after HIFU ablation. In the current study, we sought to determine whether HIFU ablation could directly increase hypoxia in the residual hepatocellular carcinoma and enhance pro-angiogenic effect through an HIF-1, 2α/VEGFA/EphA2-dependent mechanism.

## Materials and Methods

### Cell Line and Experimental Animals

HepG2 cells, a human hepatoma cell line, was brought from Cell Resource Center, Chinese Academy of Medical Sciences, Peking Union Medical College, and cultured in Dulbecco’s modified Eagle’s with high glucose supplement (DMEM) containing 10% fetal bovine serum (FBS) in a humidified incubator at 37°C with an atmosphere of 5% CO_2_. Viability of HepG2 cells determined by trypan blue exclusion was >95%. Homogenous nude mice (male athymic BALB/c nu/nu) (4–6 weeks old) were purchased from the Animal Center of Chongqing University of Medical Science. All animals received humane care in accordance with the National Institutes of Health Guidelines and the legal requirements in China. The protocol was approved by the Committee on the Ethics of Animal Experiments of the Chongqing University of Medical Science.

### Instrument and Antibodies

A focused ultrasound tumor therapeutic system (Seapostar) was provided by Chongqing Haifu (HIFU) Technology Co. Mouse monoclonal anti-HIF-1α, rabbit polyclonal anti-HIF-2α, and mouse monoclonal anti-VEGFA were purchased from Abcam (UK). DMEM, 0.25% trypsinase, and FBS were purchased from Hyclone (USA). Rabbit anti-CD31, and anti-EphA2 antibodies were purchased from Bioworld (USA), Bioss (Beijing, China), respectively.

### Subcutaneously Transplanted Tumor Models and HIFU Ablation

HepG2 cells were inoculated subcutaneously (s.c.) into the right flank of the mice (5×10^6^ cells per mouse in 0.2 ml). When the tumors reached 1.5–2.0 cm, animals were treated with Seapostar therapy at 8.6 MHz, 5 w, 30 s, and repeated leaving about 10% residual tumor tissue (measured by computed tomography (CT) scan) to simulate clinical tumor recurrence after HIFU. All athymic BALB/c nu/nu mice were anesthetized with 30 mg/kg pentobarbital. The mice were divided randomly into seven groups according to points after treatment (1st, 3rd, 5th day and 1st, 2nd, 3rd, 4th week) and control group (no treatment). Each group contained six mice (except the control group, and the 4^th^ week group which contained five mice in each). Two mice died during treatment, and were not assigned to any group.

### Tissue Preparation

The mice were anesthetized with pentobarbital prior to sacrifice by cervical dislocation. Tumors were harvested at various time, and samples from each group were snap-frozen in liquid nitrogen for RNA and protein preparation. Corresponding tissue samples were fixed in 4% formalin for paraffin-embedded sections.

### Immunohistochemistry and Microvascular Density Assay

The paraffin-embedded tissues were cut into 4 µm sections. Slides were dewaxed and hydrated. Endogenous peroxidase was blocked with 3% hydrogen peroxide for 20 min and non-specific binding was blocked with goat serum (10%) in PBS for 20 min. The slides were incubated with anti-HIF-1α (1∶200), anti-HIF-2α (1∶2500), anti-VEGFA (1∶50), anti-EphA2 (1∶100) and anti-CD31 (1∶50) at 4°C overnight. After washing, the slides were incubated with horseradish peroxidase-labeled second antibody at 37°C for 20 min. Finally, they were incubated in phosphate buffered saline containing diaminobenzidine (DAB) for 5 min and then examined on a microscope.

The intensity of immunohistochemical staining was evaluated in five areas of each section. All samples were reviewed by two independent investigators including a pathologist, who were blinded to the experimental groupings. Points for percentage of positive cells, and the intensity were combined, and an overall score index (SI 0–3) was assigned. Briefly, the percentage of positively stained cells was rated as: 0 (0–5%); 2 (6–50%); 3 (>50%). The staining intensity was graded as follows: 1 point, weak intensity; 2 points, moderate intensity; 3 points, strong intensity. Tumors were categorized into four grades based on the SI: negative expression SI, 0 or <5% cells stained regardless of intensity; weak expression (SI, 1) 1 to 2 points; moderate expression (SI, 2) 3 to 4 points; strong expression (SI, 3) 5 to 6 points [13]. The specimens of grade 3 and 4 were recorded as positive results in the statistical analysis.

Microvascular density (MVD) was determined according to the criteria introduced by Tian et al [14]. Briefly, the areas of highest CD31-positive vessel density were screened at ×40 magnification, and then counted at ×200 magnification in 10 random fields. The mean number of micro-vessels in each field was determined and expressed as the MVD.

### Western Blot Analysis

Protein extracts were obtained using a protein extraction kit. Protein concentration was determined by the Bradford assay kit (Bio-Rad, Hercules, CA). The protein extract was electrophoresed on a sodium dodecyl sulphate - polyacrylamide (SDS - PAGE) gel and transferred to polyvinylidene fluoride (PVDF) membranes. After incubation with 5% dry non-fat skimmed milk to block non-specific binding, the membranes were exposed to specific anti-HIF-1α (1∶500), anti-HIF-2α (1∶1000), anti-VEGFA (1∶200), anti-EphA2 (1∶100), and anti-β-actin (1∶1000, Santa Cruz Biotechnology) monoclonal antibodies overnight at 4°C. The membranes were washed and exposed to peroxidase-conjugated anti-IgG secondary antibody (1∶5000). Finally, the immune complexes were developed using an enhanced chemiluminescence detection kit according to the manufacturers instructions (Pierce, Waltham, MA) and the GelGDoc2000 imaging system (Bio-Rad Germany) was employed to analyze the bands, and the protein levels by the relative optical density.

### Quantitative RT-PCR Analysis

Total RNA was isolated from tissues using an SV total RNA isolation kit (Promega, USA) according to the manufacturer’s instructions. The forward primer for HIF-1α was: 5′ - AAACCTAAATGTTCTGCCTAC - 3′ and the reverse: 5′- GGATGTTAATAGCGACAAAGT - 3′. The forward primer for HIF-2α was: 5′ - GCACCAAGGGTCAGGTAGTAAG - 3′ and the reverse: 5′ - CAGGTTGCGAGGGTTGTAGAT - 3′. The forward primer for VEGF-A was 5′ - AGGGAAGAGGAGGAGATGAGA - 3′ and the reverse: 5′ - GGCTGGGTTTGTCGGTGTT- 3′. The forward primer for EphA2 was 5′ - GCAAAGGGTGGGACCTGATG - 3′ and the reverse: 5′ -TTGGTGCGGAGCC -. AGTTGT - 3′. The samples were incubated at 70°C for 5 min, chilled on ice, and then reverse-transcribed into cDNA using a TIANGEN assay kit. The mixture was incubated at 42°C for 20 min, 99°C for 5 min, 4°C for 5 min to deactivate reverse transcription. PCR was performed in a 20 µL final volume containing H_2_O up to 20 µL, 1 µL cDNA diluted in RNase-free water, 10 µL SYBR premix ex-Taq, and antisense and sense primer (10 µmol/L, 0.5 µL each). The sample was heated to 95°C for 2 min in the initial denaturation step, followed by amplification for 40 cycles at 95°C for 10 s, the annealing temperature for 15 s, and 72°C for 45 s, and 1 cycle at 72°C for 10 min. The β-actin was used for internal competitive reference standard, the comparative ct (threshold cycle) method was used to calculate the relative changes in gene expression using the value of 2 ^− ΔΔCT^.

### Statistical Analysis

Data were analyzed using SPSS 10.0 software and expressed as the mean ± SD (±s). Through inspection (p>0.05), the sample data were found to satisfy homogeneity of variance. Statistical analysis was carried out by one-way ANOVA. If the type I error was assumed to be 0.05, and the standard deviation (sd = 0.2), with a statistical power of 0.8, the minimum sample size required was 40. Therefore, in this study, 48 mice were considered to be adequate. P values of <0.05 were considered to be statistically significant.

## Results

### Residual Tumor Tissue and Histochemical Staining

The residual hepatic tumor tissue after HIFU treatment was found to be grayish white in color with a complete capsule, a fish flesh-appearing cut surface, and partial central liquefaction with a necrotic appearance (Swiss cheese). The histopathological features noted on (HE) were necrosis and infiltration by inflammatory cells in surrounding areas (Figure 1).

**Figure 1:** The picture shows residual hepatic tumor tissue after high intensity focused ultrasound (HIFU) treatment. (**a**) The residual hepatic tumor tissue was obtained from the subcutaneously transplanted tumor. (**b**) The cut surface of the residual tumor tissue. (**c**) Residual tumor tissue with hematoxylin and eosin staining, revealing necrotic cells (**d**), inflammatory cells (**e**), and normal hepatoma cells (**f**). Original magnification, ×200. Scale bars: 20 µm.

### Immunohistochemical Staining of HIF-1, 2α, VEGFA, and EphA2

HIF-1, 2α, VEGFA, and EphA2 protein were predominantly localized to the cytoplasm of the cells. The brown-yellow or dark brown staining of the cytoplasm was considered positive. Compared to the control group, the greatest expression of HIF-1α was on the 3rd day (Figure 2). However, the highest expression of HIF-2α protein was on the 2nd week (P<0.01) (Figure 3). Compared to the control group, VEGFA and EphA2 protein expression were markedly decreased from the 1st day to the 1st week (P<0.01), and increased from the 2nd week to the 4th week (Figure 4, Figure 5).

**Figure 2:** An immunohistochemistry analysis of hypoxia inducible factor-1α (HIF-1α). Controls (a), HIF-1α protein expression on the 3rd day (c vs a, b, f, g, h) (P<0.01), and subsequent time points (b vs e, and a vs f, g, h, P>0.05). Original magnification, ×200. Scale bars: 20 µm.

**Figure 3:** An immunohistochemistry analysis of hypoxia inducible factor-2α (HIF-2α). Control group (a), HIF-2α protein levels on the 2^nd^ week (f vs a, b, c) (P<0.01), and the 2^nd^ to 4^th^ week (P<0.05). Original magnification, ×200. Scale bars: 20 µm.

**Figure 4:** An immunohistochemistry analysis of vascular endothelial growth factor A (VEGF-A). Control group (a), HIFU treatment from the 1st day to the 1st week (b, c, d, e) (P<0.01), and from the 2st week to the 4st week (a vs h, P<0.05). Original magnification, ×200. Scale bars: 20 µm.

**Figure 5:** The immunohistochemistry analysis of epithelial cell kinase (EphA2). Control group (a), EphA2 protein levels from the 1st day to the 1st week (b, c, d, e) (P<0.01), and from the 2nd week to the 4th week (a vs h P<0.05). Original magnification, ×200. Scale bars: 20 µm.

The expression of CD31, an indicator of intra-tumoral MVD, was extremely low (1 d–1 w), but significantly increased (2–4 weeks) compared with the control group (P<0.01) (Figure 6). The expression patterns of VEGF-A, EphA2, and MVD were similar (P<0.05) (Figure 7).

**Figure 6:** MVD analyses. Control group (a), micro-vessel density (MVD) from the 1^st^ day to the 1^st^ week (b, c, d, e) (P<0.01), and from the 2nd week to the 4th week (g vs a, P<0.05). Original magnification, ×200. Scale bars:20 µm.

**Figure 7:** The expression level of VEGFA and EphA2 protein, and MVD counts detected by immunohistochemistry as a function of time. (vs. each other, coefficient of correlation = 0.981, *P*<0.01).

### Western Blot Analysis of the Expression of the HIF-1, 2α, VEGF-A, and EphA2 Protein in Residual Tumor Tissues

HIF-1α protein levels were significantly increased in the 3rd group, compared with the other groups (except on the 5^th^ day) (P<0.01). There was no significant difference between levels on the 1^st^ day and the 1^st^ week (P>0.05), also among control groups, or levels on the 2^nd^, the 3^rd^, and the 4^th^ week compared with each other (P>0.05) (Figure 8). The expression of HIF-2α protein was significantly higher in the 2nd week compared with the control group (p<0.01), and continued at a high level from the 2nd week to the 4th week and then decreased slowly (Figure 9). Compared with control group, the expression of VEGF-A and EphA2 protein decreased rapidly from 1 d to 1 w (P<0.01), then increased gradually from 2 w to 4 w (P<0.05). However, there was no statistical significance between levels on the 2nd week and control group (P>0.05) (Figure 10).

**Figure 8:** HIF-1α protein expression on the 3^rd^ day, compared with the control group and other groups of the time points (P<0.01). (1^st^ day vs the 1^st^ week, P>0.05, from the 2 w to 4 w group, compared with each other, P>0.05).

**Figure 9:** The HIF-2α protein levels on the 2^nd^ week, compared with the control group (P<0.01), from the 2^nd^ to 4^th^ week ( P<0.05, compared with the control group).

**Figure 10:** The VEGFA and EphA2 protein expression after HIFU treatment from 1 d to 1 w, compared with the control group ( P<0.01) and from the 3 w to 4 w compared to the control group, respectively (P<0.05). (2nd week vs control group, P>0.05).

### HIF-1, 2α, VEGF-A, and EphA2 mRNA Expression in Residual Tumor Tissues

The HIF-1α mRNA expression significantly was increased on the 3rd day compared with the control group (P<0.01), then decreased from 5 d to 4 w (P<0.05). There was no statistical difference between levels on the 1^st^ day and the 1^st^ week (P>0.05). However, the levels of HIF-2α mRNA were obviously increased on the 2nd week compared with other groups (P<0.01). There were no significant differences at 5d, 1w, 3w, and 4w among each other (P>0.05). The levels of VEGFA and EphA2 mRNA decreased from 1 d to 1 w (P<0.01), and then increased from 2 w to 4 w, compared to control group (P<0.05). There was no significant difference between levels of the control group and the 2nd week group (P>0.05) (Figure 11).

**Figure 11:** Hypoxia inducible factor-1, 2α, VEGFA, and EphA2 mRNA expression measured by Q-PCR. HIF-1α mRNA expression at the 3^rd^ day (P<0.01), compared with the control, and other groups of the time points (P<0.05). HIF-2α mRNA at the 2^nd^ week (P<0.01) and levels of VEGFA and EphA2 mRNA at various time points from the 1st day to the 1st week, P<0.05, and from the 3 w to 4 w, P<0.05, compared with control group, and the 2nd week vs the control group, P>0.05.

## Discussion

The phenomenon of rapid growth of residual liver tumor after HIFU ablation has been observed in many clinical centers. A previous study demonstrated that residual tumor was characterized by proliferation, invasion and metastasis when the local ablative temperature was not sufficiently high [15]. Forkman et al reported that the generation of a tumor mass required tumor cell proliferation plus angiogenesis. Tumor cell proliferation alone, in the absence of angiogenesis, gave rise to dormant, microscopic tumors of 1 mm^3^ or less. However, these in situ cancers were harmless to the host [16]. HCC is also a highly vascular tumor, and angiogenesis plays a considerable role in its development and progression [14]. Similarly, the current study revealed that angiogenesis of residual hepatocellular carcinoma after HIFU ablation was higher than that in the original carcinoma tissue.

HIF-1α is a transcription activator of the VEGF promoter. However the VEGF, whose most important member is VEGF-A, is the most potent angiogenic factor and plays a key role in tumor associated angiogenesis and hyper-permeability [8], [17], [18]. Perpetual blood vessel formation and angiogenesis are hallmarks of cancer, and prerequisites for three-dimensional tumor growth, invasion and metastasis [19]. Hypoxia induces HIF-1α, and promotes the expression of VEGF-A, the main pro-angiogenic hypoxia induced gene [20]. On the contrary, numerous studies have shown that suppression of VEGF and HIF-1α inhibit carcinoma cell proliferation [21]–[24]. These results demonstrate that HIF-1α exerts a regulatory effect on tumor angiogenesis. These studies also showed that the angiogenesis induced by HIF-1α/VEGF-A produced by altered cells after hyperthermia treatment may play an important role in the rapid growth of residual HCC after radiofrequency ablation [25].

According to our studies, we found that HIF-1α promoted residual tumor angiogenesis before the 1st week, and VEGF-A expression was increased. These results are in good agreement with previous findings. However, the mediating effects of HIF-1α were reduced from the 2nd week to the 4th week compared with original cancerous tissue group. On the contrary, the levels of HIF-2α protein and mRNA were weaker than HIF-1α expression levels before the 1st week after HIFU treatment. The expression of HIF-2α and VEGF-A was increased from the 2nd week to the 4th week, which promoted tumor angiogenesis. The alteration of VEGF-A, EphA2 expression, and MVD were coincident with the trends of HIF-1α and HIF-2α. These results suggested that residual tumor angiogenesis was regulated by HIF-1α and HIF-2α at different time points and mechanisms. It is possible that they promoted each other or acted independently.

From the previous discussion, there are several possible explanations for this phenomenon: low O_2_ and other stresses associated with tumor growth activate p53, a critical tumor suppressor that is mutated or silenced in a majority of human cancers [26]. Numerous studies have shown that p53 accumulation occurs within hypoxic regions of solid tumors, and correlates with cells undergoing apoptosis [27]. MDM2 over-expression actually promotes p53 accumulation and target gene stimulation when HIF-1α is activated in hypoxic cells [28]. Furthermore, HIF-1α appears to enhance p53 activation by ionizing radiation, resulting in increased p53 phosphorylation and p53-mediated apoptosis [29]. It should also be noted that there is a lack of balance between HIF-1α and p53, a potential negative feedback loop for HIF-1α activity in HCC after HIFU. This may enhance residual tumor hypoxia. We assume that HIF-1α is the most prominent activator of p53. Therefore, the current results demonstrated that HIF-1α increased VEGF-A expression, but residual tumor angiogenesis was not substantial from the 1st day to the 1st week.

Pahlman et al first demonstrated that HIF-2α protein is stabilized at moderate (2–5% O_2_) levels, whereas HIF-1α accumulated only at lower (0–2% O_2_) levels in HeLa and neuroblastoma cells [30], [31]. This means that HIF-2α accumulates at higher O_2_ levels than HIF-1α, which may allow its selective activation in blood vessels. The level of HIF-1α protein and mRNA increased rapidly upon hypoxic exposure, but then declined after several days. In the current study, the levels of HIF-1α protein and mRNA in residual tumor tissues decreased gradually, while residual tumor angiogenesis and oxygen concentration increased (1 w–4 w). However, the levels of HIF-2α protein and mRNA were increased. HIF-2α expression is more restricted, and particularly abundant in blood vessels [32]. This observation led to the hypothesis that the primary role of HIF-2α was to modulate vascular endothelial cell function, an idea supported in part by the close correlation of HIF-2α and VEGF mRNA expression patterns [33]. Thus, the expression of VEGF-A protein and mRNA were increased higher after 2 w – 4 w, with an increase in microvessel density of residual tumor.

EphA2, a receptor tyrosine kinase and a member of the Eph (ephrin­receptor) family of PTKs, has been found to play an important role in angiogenesis [34], [35]. Further supporting the role of EphA2 in angiogenesis is a study by Cheng et al, where treatment of transgenic mice with soluble EphA2 receptors resulted in enhanced endothelial cell apoptosis in an orthotopic pancreatic cancer model [36]. Moreover, it is well established that the Eph system promotes tumor angiogenesis. EphA2 supports cancer progression. Tumors with EphA2 over-expression were significantly associated with high levels of angiogenesis markers, specifically VEGF-A expression and MVD counts. Furthermore, EphA2 kinase function in the tumor microenvironment seemed to be necessary not only for tumor angiogenesis, but also for metastatic progression [37]. Tumor cells that over-express EphA2 are involved in vascular mimicry (VM) and form vasculogenic-like networks in vitro, thus affecting tumor cell plasticity [38]. It could be concluded PTKs (especial EphA2) are pivotal factors of VM. Based on these data, it was deduced that EphA2 not only promoted angiogenesis of residual tumor (2 w–4 w), but also provided the prerequisite conditions for the angiogenesis, growth, and metastasis of residual tumor earlier than the process of angiogenesis. In this study, the change in EphA2 and VEGF-A levels were basically simultaneous. Research has shown that VEGF may significantly stimulate EphA2 and VE­cad expression at the protein and mRNA levels in ovarian tumor cells. MMP­2 and MMP­9 which act as effecter molecules, induced by EphA2, are controlled by VEGF [39], and HIF-1α gene silence can suppress the growth of esophageal squamous cancer in vivo and inhibit the EphA2 and VE-cadherin expression in the formation of vasculogenic mimicry. HIF-1α may participate in the regulation of vasculogenic mimicry through these two sites in esophageal squamous cancer [40]. Hypoxia has also been shown to induce VM in hepatocellular carcinoma, and induce the formation of VM channels to acquire an adequate blood supply [41]. Several key molecules, including VE-cadherin, matrix metalloproteinases, laminin-5γ2 chain, and EphA2 have been implicated in VM. Moreover, studies have shown that HIF-1α expression induces the formation of VM channels to acquire an adequate blood supply [42]. Thus, developing treatment strategies that target EphA2 could also provide novel alternative options for patients with HCC after HIFU treatment.

These results indicated that HIF-1α and HIF-2α promoted tumor angiogenesis, and acted complementarily at various time points. We postulated that HIFU led to residual tumor tissue due to its pro-angiogenic effect through enhancement of the HIF-1, 2α/VEGF-A/EphA2 signaling pathway. These novel findings could be a potential mechanism associated with the rapid growth of the residual tumor after HIFU ablation and, therefore, could have important therapeutic implications.

Although HIF-1α and HIF-2α share numerous target genes, and highly conserved structural features, mounting evidence indicates that each protein has remarkably distinct functions in specific cellular contexts, which are mediated in part by regulation of unique target genes, including c-Myc [43], p53 [44], and nitric oxide [45]. HIF-1α and HIF-2α have different and largely non-overlapping functions in pathophysiological angiogenesis. For instance, hypoxic VEGF expression is driven primarily by HIF-1α in ECs, whereas hypoxic Dll4 and Ang2 expression are regulated primarily by HIF-2α, suggesting an important division of transcriptional labor that underlies the complementary effects on EC behavior. Namely, HIF-1α promotes EC proliferation, growth, and morphogenesis in response to local hypoxic stress. However, these activities are fine-tuned and restrained by HIF-2α to promote vessel remodeling and produce a mature, functional vascular network [46]. All these are consistent with observed mechanisms of HIF-1, 2α in angiogenesis, development, invasion and metastasis of residual tumor after HIFU treatment. This will likely become an important field, and the identification of regulating mechanisms could provide novel targets for anti-angiogenic cancer therapies.

In conclusion, to the best of our knowledge, this is the first study to investigate the clinical and molecular biology correlates between HIF-1, 2α expression and angiogenesis in HCC. Our findings were that HIFU ablation likely enhanced the hypoxia condition of residual tumor, due to tumor angiogenesis via HIF-1, 2α/VEGFA/EphA2. This is the underlying mechanism and a potential therapeutic target of the rapid growth of residual HCC. Furthermore, these results indicated that HIF-1α and HIF-2α are viable targets, alone or in conjunction with anti-angiogenic (anti-VEGF-A or anti-EphA2 drug) cancer therapies, for the treatment of patients with HCC after HIFU ablation. However, further research is needed to clarify the underlying molecular mechanism of rapid growth of residual HCC after HIFU treatment.
